# Circ_0001998 Regulates the Proliferation, Invasion, and Apoptosis of Lung Adenocarcinoma via Sponging miR-145

**DOI:** 10.1155/2022/6446150

**Published:** 2022-05-11

**Authors:** Qiang Shi, Jian-Gang Ju

**Affiliations:** ^1^Department of Thoracic Surgery, Hwa Mei Hospital, University of Chinese Academy of Science, Ningbo, Zhejiang, China; ^2^Department of Respiratory, First People's Hospital of Linping District, Hangzhou, Zhejiang, China

## Abstract

Circular RNA (circRNA) is considered an important regulator of cancer. Circ_0001998 is a newly discovered circRNA and its role in lung adenocarcinoma (LUAD) remains obscure and requires further study. The expression levels of circ_0001998 and miR-145 in LUAD were predicted by bioinformatics analysis and then verified by qRT-PCR in the LUAD cell lines. CCK-8, clone formation, EdU assay, and flow cytometry were applied to determine the effects of silencing circ_0001998 on the viability, proliferation, and apoptosis of LUAD cells. The target relationship between circ_0001998 and miR-145 was predicted by bioinformatics analysis and verified by a luciferase activity experiment. The effect of circ_0001998/miR-145 axis on the viability, proliferation, and apoptosis of LUAD cells was verified by the rescue experiment. Circ_0001998 was upregulated in LUAD, and silencing circ_0001998 suppressed viability, proliferation, and invasion of LUAD cells. The target gene of circ_0001998, miR-145, was downregulated in LUAD, and the low expression of miR-145 indicated a poor prognosis. The effect of silencing circ_0001998 on the biological function of LUAD cells was reversed by the miR-145 inhibitor. Circ_0001998 regulates the proliferation, invasion, and apoptosis of LUAD via sponging miR-145.

## 1. Introduction

Lung cancer is the most common malignant tumor in the world. From the perspective of pathology, lung cancer can be divided into nonsmall cell lung cancer (NSCLC) and small cell lung cancer, in which NSCLC accounts for about 85% of lung cancer [1]. As the most common subtype of NSCLC, the incidence rate of lung adenocarcinoma (LUAD) in lung cancer incidence rate is 40%, and it has been increasing obviously in the past decades [2]. In retrospect, surgery, radiotherapy, and chemotherapy were the three traditional methods of treating lung cancer. However, with the deepening of cancer research, the limitations of these three treatment methods have gradually emerged. Hence, it is still an important task to find new and effective diagnosis and treatment methods for LUAD.

In recent years, with the vigorous development of molecular biotechnology, circular RNA (circRNA) has become a research hotspot, providing a new direction for tumor research [3]. The circRNA is different from linear RNA, and its closed-loop molecular structure makes it less susceptible to the influence of ribonuclease R (RNase R), so its expression is more stable [4]. At present, mounting evidence showed that circRNA is closely engaged in the proliferation, invasion, and apoptosis of multiple tumor cells, including LUAD, which is expected to become a therapeutic target or prognostic marker of cancer [5–7]. Circ_0001998, a newly discovered circRNA, is derived from the FUT8 (fucosyltransferase 8) gene, which may be related to the development of colorectal cancer [8], but its role in LUAD has not been reported.

One of the important functions of circRNA is to adsorb miRNAs like a sponge, thereby preventing miRNAs from inhibiting the expression of their target genes [9]. This mechanism has been found to be widespread in LUAD. For example, Wang et al. pointed out that circRNA-002178 adsorbed miR-34 to regulate the immune escape of LUAD [10], Zhou et al. revealed that the circRNA-ENO1/miR-22-3p/ENO1 axis engaged in the glycolysis process of LUAD [11], and Xu et al. found that circ_0000326 acts as a sponge of miR-338-3p and exacerbates the deterioration of LUAD [12].

Through preliminary experiments, we found that circ_0001998 is upregulated in LUAD. This suggests that circ_0001998 is likely to implicate the development of LUAD. Therefore, this article will explore the possible mechanism of circ_0001998 in LUAD.

## 2. Materials and Methods

### 2.1. Bioinformatics Analysis

The expression profile of circRNA related to lung cancer (GSE112214 and GSE101586) was downloaded from the GEO database. The target miRNA of circ_0001998 was screened through the Circular RNA Interactome database, StarBase, and downregulated miRNAs in GSE74190 and GSE63805 datasets. The GEO datasets (GSE74190 and GSE63805) were used to compare the expression levels of hsa-miR-145 in tumor tissues and nontumor tissues. The overall survival curve of LUAD patients with low and high hsa-miR-145 expression was examined by the Kaplan–Meier plotter.

### 2.2. Cell Culture

Human immortalized lung epithelial cells BEAS-2B and human LUAD cell lines (HCC827, H460, H1975, A549, and H1299) purchased from Cell Bank of the Chinese Academy of Science (Shanghai, China) and grown in Roswell Park Memorial Institute (RPMI)-1640 medium (72400120, Gibco, USA) supplemented with 10% fetal bovine serum (FBS) (10091, ThermoFisher, USA) and 1% penicillin-streptomycin (15140-122, ThermoFisher, USA) in 37°C, 5% CO_2_ incubator (Forma Steri-Cycle, Thermo Scientific, USA).

### 2.3. Transfection

Si-Circ_0001998-1 (5′-ATCTCTCCGGTTGCTGCTTTT-3′), si-Circ_0001998-2 (5′-GAATCTCTCCGGTTGCTGCTT-3′), and si-Circ_0001998-3 (5′-AATCTCTCCGGTTGCTGCTTT-3′) were synthesized by Sangon Company. miR-145 mimic and inhibitor were purchased from RiboBio Company (Shanghai, China). The transfection step was assisted by Lipofectamine 3000 (L300008, ThermoFisher, USA). 24 hours after transfection, the transfection efficiency was determined by the quantitative reverse transcription-polymerase chain reaction (qRT-PCR).

### 2.4. qRT-PCR

To determine mRNA expressions, total RNA was extracted from cells by the total RNA extraction kit (DP419, TIANGEN, China). Subsequently, the complementary DNA from each sample was synthesized by reverse transcription reactions using a reverse transcription kit (D7166, Beyotime, China). The qRT-PCR was conducted by a real-time PCR system (7300, Applied Biosystems, USA) with SYBR Green qPCR Mix (D7260, Beyotime, China) as per the guide. The primers are given in Table 1. The expression levels of circ_0001998-1 and miR-145 were normalized to glyceraldehyde-3-phosphate dehydrogenase (GAPDH) or U6 expression by the 2^−ΔΔCt^ method.

### 2.5. Cell Viability

In order to evaluate the viability of the cells after transfection, we conducted cell viability experiments by the Cell Counting Kit-8 (CCK-8) (M4839, AbMole, China). First, the cells were seeded in 96-well plates. When the fusion degree of cells reached about 80%, CCK-8 solution was added to the well and incubated for 2 hours. The absorbance at 450 nm was measured with a microplate reader (SpectraMax5, Molecular Devices, USA).

### 2.6. Colony Formation Assay

Colony formation assay was performed on A549 and H1299 cells transfected with or without si-circ_0001998-1 for assessing proliferative capacity. The cells were collected and resuspended in a 6-well plate at a density of 5 × 10^2^ per well and incubated for 2 weeks. Afterwards, the indicated cells were washed with phosphate-buffered saline (C0221A, Beyotime, China), treated with 4% paraformaldehyde (P1110, Solarbio, China) and stained by crystal violet dying (C196471, Aladdin, China). The final colony numbers of cells were observed by an inverted microscope (DM2700P, Leica, Germany).

### 2.7. 5-Ethynyl-2′-deoxyuridine (EdU) Assay

The Yefluor 594 EdU Imaging Kit (40276ES60, YEASEN, China) was employed to determine the proliferative capacity of A549 and H1299 cells transfected with or without si-circ_0001998-1. In short, the cells were seeded in a 96-well plate and cultured for 24 hours. The EdU working solution was added to 96-well plates and continued to incubate for 2 hours. After incubation, the cells were treated with 4% polyformaldehyde, 0.5% Triton X-100 (A600198, Sangon, China), and click-iT reaction mixture, respectively. DAPI staining solution (E607303, Sangon, China) was used to stain the nucleus, and then, fluorescence was detected by the fluorescence microscope (E800, Nikon, Japan) after washing.

### 2.8. Apoptosis Assay

The Annexin V-FITC Apoptosis Detection Kit (C1062S, Beyotime, China) was performed to determine the cell apoptosis rate. Cells were stained with Annexin V-FITC and propidium iodide for 20 minutes at 25°C in dark following the protocol. At last, the stained cells were collected and analyzed by a flow cytometer (Cytoflex3L8C, Beckman, USA).

### 2.9. Transwell Assay

A transwell experiment was used to evaluate the invasion ability of A549 and H1299 cells after transfection. Cells need to be deprived of serum culture before the invasion experiment. Then, cells were added into transwell inserts (353097, Corning, USA) which were coated with Matrigel (354480, Corning, USA). Meanwhile, the medium containing 10% FBS was injected into the lower chamber as a chemoattractant. After culturing for 24 hours, a cotton swab was employed to remove noninvaded cells adhering on the upper surface, while the invaded cells were subject to paraformaldehyde and crystal violet treatments. The invasion of A549 and H1299 cells were observed by an optical microscope.

### 2.10. Luciferase Activity Assay

The relationship between circ_0001998 and miR-145 was confirmed by the dual-luciferase reporter assay system (E1910, Promega, USA). The complementary fragments of circ_0001998 and miR-145 were amplified and cloned into the psiCHECK-2 vector (TB329, Promega, USA), named circ_0001998-WT (wild-type). A mutant type (MUT) of circ_0001998 was also constructed and named circ_0001998-MUT. miR-145 mimic, miR-145 negative control (NC), and these vectors were cotransfected into cells by Lipofectamine 3000 for 24 hours. After that, the luciferase activity was measured by the Cellometer Auto 2000 Cell Viability Counter (Nexcelom, USA).

### 2.11. Statistical Analysis

Data were analyzed by Graph Prism v8.0 (GraphPad Software, California, USA) and represented as mean ± standard deviation. An independent sample *t*-test was used for comparison between two groups. Differences between multiple groups were analyzed by a one-way analysis of variance. *P* < 0.05 was accepted to be statistically significant.

## 3. Results

### 3.1. Circ_0001998 Was Upregulated in LUAD

Based on the expression profiles of lung cancer-related circRNAs in the GEO database (GSE112214 and GSE101586), we screened the upregulated or downregulated circRNAs in LUAD and then crossed them to obtain 7 upregulated circRNAs and 4 downregulated circRNAs (Figures 1(a)–1(c)). According to the results of the heat map, we selected circ_0001998 as the research object (Figure 1(d)). After that, we verified by qRT-PCR that the expression of circ_0001998 in LUAD cell lines is much higher than that of lung epithelial cells BEAS-2B (Figure 2(a), *P* < 0.05). Because circ_0001998 is expressed relatively higher in A549 and H1299 cells, we chose these two cell lines for follow-up experiments.

### 3.2. Silent circ_0001998 Inhibited Tumor Growth In Vitro and In Vivo

We designed three siRNAs to specifically silence circ_0001998. According to the results of qRT-PCR (Figure 2(b), *P* < 0.05), the inhibitory effect of si-circ_0001998-1 is the best in both cell lines, so we selected si-circ_0001998-1 for follow-up experiments. CCK-8 experiment proposed that si-circ_0001998-1 transfection for 48 h, 72 h, and 96 h repressed the viability of A549 and H1299 cells (Figure 2(c), *P* < 0.05). The relative colony formations were attenuated in the si-circ_0001998-1 group compared with the si-NC group (Figure 3(a), *P* < 0.01). Moreover, silent circ_0001998 suppressed the proliferation (Figure 3(b), *P* < 0.05) and invasion (Figure 4(b), *P* < 0.01), but elevated apoptosis (Figure 4(a), *P* < 0.01) of A549 and H1299 cells.

### 3.3. Circ_0001998 Targeting miR-145 to Regulate the Vitality, Proliferation, and Invasion of LUAD Cells

We analyzed the possible target genes of circ_0001998 through bioinformatics analysis and then took the intersection to obtain that miR-145 is a possible target gene of circ_0001998 (Figure 5(a)). GEO datasets (GSE74190 and GSE63805) showed that hsa-miR-145 was upregulated in tumor tissues compared to that in nontumor tissues (Figure 5(b)). In addition, the overall survival curve of LUAD patients with low and high miR-145 expression showed that patients with low miR-145 have a poorer prognosis than those with high miR-145 (Figure 5(c)).

Figure 6(a) shows the predicted binding sites of circ_0001998 and miR-145. The binding relationship between the two was verified by the dual-luciferase reporter gene experiment, that is, miR-145 mimic suppressed the luciferase activity in the circ_0001998-WT group instead of the circ_0001998-MUT group (Figures 6(b)-6(c), *P* < 0.01). Significant downregulation of miR-145 can be observed in H460, A549, and H1299 cells, but the miR-145 expression in HCC827 and H460 is not significantly different from that in BEAS-2B (Figure 6(c), *P* < 0.05). Silencing circ_0001998 in A549 and H1299 cells can promote the expression of miR-145, but miR-145 inhibitor can reverse the promotion effect of si-circ_0001998-1 (Figures 6(d)-6(e), *P* < 0.01). 72 h after si-circ_0001998-1 transfection, the inhibitory effect of the miR-145 inhibitor on cell viability caused by si-circ_0001998-1 began to appear, but the inhibitory effect of the miR-145 inhibitor changed significantly only 96 hours after H1299 cells transfected with si-circ_0001998-1 (Figure 7(a), *P* < 0.01). Additionally, the inhibitory effect of silent circ_0001998 on cell proliferation and invasion was also overturned by the miR-145 inhibitor (Figures 7(b)-7(c), *P* < 0.01).

## 4. Discussion

Traditional Chinese medicine (TCM) and its natural products relieve adverse effects and enhance the efficacy of radiotherapy and chemotherapy in the cancer treatment. However, the anti-LUAD mechanisms of Chinese herbal medicines and their bioactive components remain largely elusive. An increasing number of studies have shown that circRNA exerts a pivotal effect in regulating tumor development. For example, Yang et al. reported that *Scutellaria barbata* D. Don (SB) and *Oldenlandia diffusa* (Willd.) Roxb may inhibit hepatocellular carcinoma cell growth in vitro and in vivo through altering circRNA-miRNA-gene expression [13]. In addition, Xu et al. showed that curcumin, discovered in *Curcuma longa*, inhibited NSCLC growth through downregulating circ-PRKCA [14]. Nevertheless, the effects and mechanism of circ_0001998 in the LUAD process are unknown. In order to reveal the regulatory mechanism of circ_0001998 in LUAD, we silenced circ_0001998 and evaluated the changes in the malignant biological behavior of LUAD cells for developing new treatment natural products to improve the prognosis of LUAD. The experimental results showed that silencing circ_0001998 hinders the development of LUAD.

We initially determined the research object as circ_0001998 through bioinformatics analysis. Like other circRNAs, circ_0001998 can be used as a sponge of miRNA to participate in the progression of cancer, which was also been confirmed in the study of the circRNA-miRNA regulatory network in colorectal cancer by Yuan et al. [8]. Therefore, we predicted and confirmed that the target gene of circ_0001998 is miR-145. Like circRNA, miRNAs are also widespread in cells, but the functions of the two are different. CircRNA mainly acts by adsorbing miRNA, while miRNA plays a regulatory role in tumors by degrading or inhibiting the translation of mRNA. The study by Zong et al. pointed out that circWHSC1 adsorbs miR-145 to promote the development of ovarian cancer [15].

miR-145 acts as an antioncogene in a variety of tumors and can inhibit the malignant biological behavior of tumors by targeting multiple oncogenes [16]. L Huang detected that the level of miR-145 in the pleural effusion of lung cancer patients was significantly lower than that in the control group, and the expression level of miR-145 was also related to lymph node metastasis and the degree of differentiation of lung cancer, suggesting that miR-145 may be a potential diagnostic indicator for lung cancer [17]. Similar to L Huang's conclusion, we also found that miR-145 is underexpressed in lung cancer cell lines. Of note, the antitumor effect of miR-145 in lung cancer has been confirmed. Liu et al. revealed that miR-145 is downregulated in NSCLC cells, and overexpression of miR-145 contributes to decreased metastasis of NSCLC cells [18]. Similarly, the study by Yin et al. also showed that miR-145 can act as an EMT inhibitor in NSCLC cells, thereby hindering the metastasis of NSCLC [19]. Li et al. pointed out that the upregulation of miR-145 increased apoptosis and decreased proliferation of NSCLC cells, while silencing miR-145 did the opposite [20]. These studies indicate that the downregulation of miR-145 is one of the causes of insufficient apoptosis and excessive proliferation of lung cancer cells.

In our study, we have confirmed through rescue experiments that circ_0001998 is involved in regulating the proliferation, invasion, and apoptosis of LUAD cells by adsorbing miR-145. Interestingly, miR-145 is not only regulated by circ_0001998 in lung cancer but also regulated by other circRNAs. Xie et al. demonstrated that circEPSTI1 adsorbs miR-145 to upregulate the expression of HMGB3, thereby accelerating the proliferation and metastasis of NSCLC [21]. Cao et al. found that circ_0102231 regulates the miR-145/RBBP4 axis to promote the proliferation and invasion of NSCLC [22]. However, our research also has shortcomings. We only verified that the circ_0001998/miR-145 axis is involved in regulating the proliferation, invasion, and apoptosis of LUAD cells, but we did not explore the specific molecular mechanism.

## 5. Conclusion

In general, our research clarified the effect of circ_0001998/miR-145 axis on the development of LUAD, providing a theoretical basis for LUAD gene therapy.

## Figures and Tables

**Figure 1:** Identification of differentially expressed circRNAs in lung adenocarcinoma (LUAD). (a) Volcano plot of the differential expressed circRNAs in the GSE112214 dataset. (b) Volcano plot of the differential expressed circRNAs in the GSE101586 dataset. (c) The downregulated and upregulated circRNAs obtained in the GSE112214 and GSE101586 datasets via Venn diagram analysis. (d) Heatmap of the 11 selected LUAD-specific circRNAs in the GSE112214 and GSE101586 datasets.

**Figure 2:** Downregulation of circ_0001998 suppressed LUAD cell vitality. (a) The expression of circ_0001998 in the LUAD cell lines measured by qRT-PCR. (b) The expression of circ_0001998 detected after transfection in A549 and H1299 cells by qRT-PCR. (c) CCK-8 assays used to detect the cell vitality of A549 and H1299 cells. ^*∗*^*P* < 0.05, ^*∗∗*^*P* < 0.01.

**Figure 3:** Silence of circ_0001998 inhibited cells proliferation. (a) Colony formation assays performed to detect the clone ability of A549 and H1299 cells after transfection. (b) The proliferation of A549 and H1299 cells detected with the EdU assay after knockdown of circ_0001998. ^*∗*^*P* < 0.05, ^*∗∗*^*P* < 0.01.

**Figure 4:** Silence of circ_0001998 promotes cell apoptosis and inhibits invasion in vitro and inhibits subcutaneous tumor growth in vivo. (a) Silence of circ_0001998 increased apoptotic cells by flow cytometry. (b) The invasion of A549 and H1299 cells transfected with si-NC or si-circ_0001998 detected by transwell invasion assay. ^*∗*^*P* < 0.05, ^*∗∗*^*P* < 0.01.

**Figure 5:** Identification of targets of circ_0001998. (a) Target miRNAs of circ_0001998 identified with the circular RNA interactome database, StarBase, and downregulated miRNAs in GSE74190 and GSE63805 datasets. (b) GEO datasets (GSE74190 and GSE63805) showed that hsa-miR-145 significantly increased in tumor tissues compared to nontumor tissues. (c) The overall survival curve of LUAD patients with low and high hsa-miR-145 expression examined by the Kaplan–Meier plotter.

**Figure 6:** Circ_0001998 functions as ceRNA for miR-145 in A549 and H1299 cells. (a) The putative binding sites for circ_0001998 and miR-145. (b) The relative luciferase activity of wild-type or mutated circ_0001998 3′-UTRs luciferase vector after transfection with or without miR-145 mimic in A549 and H1299 cells. (c) qRT-PCR analysis for the expression levels of miR-145 in LUAD cell lines. (d) qRT-PCR analysis of the miR-145 expression in A549 and H1299 cells transfected with si-NC and si-circ_0001998, respectively. (e) qRT-PCR analysis of the miR-145 expression in A549 and H1299 cells transfected with miR-145 inhibitor together with si-circ_0001998, respectively. ^*∗*^*P* < 0.05, ^*∗∗*^*P* < 0.01.

**Figure 7:** miR-145 inhibition reversed the effects of si-circ_0001998 on A549 and H1299 cells. (a, b) The cell proliferation of A549 and H1299 cells transfected with miR-145 inhibitors and si-circ_0001998 detected by CCK-8 and clone assays, respectively. (c) Transwell assays used to measure cell invasion of A549 and H1299 cells. Data are presented as means ± SD, *n* = 3. ^*∗*^*P* < 0.05, ^*∗∗*^*P* < 0.01.

**Table 1:** Primers for quantitative real-time PCR analysis.

Gene	Forward primer (5′-3′)	Reverse primer (5′-3′)
Circ_0001998	TTCCTGGCGTTGGATTATGCT	CAAAAGCAGCAACCGGAGAGA
GAPDH	CAATGACCCCTTCATTGACC	TTGATTTTGGAGGGATCTCG
hsa-miR-145	GTCCAGTTTTTCCCAGGAATCCCT	GCTGTCAACGATACGCTACCTA
U6	CTCGCTTCGGCAGCACA	ACGCTTCACGAATTTGCGT

## Data Availability

The datasets used and/or analyzed during the current study are available from the corresponding author upon request.
